The article "Minimally invasive versus open surgery for acute Achilles tendon rupture: a systematic review of overlapping meta-analyses" was retracted in 2018. Reasons: plagiarism; overlap with other authors' work.

# Minimally invasive versus open surgery for acute Achilles tendon rupture: a systematic review of overlapping meta-analyses

**DOI:** 10.1186/s13018-016-0401-2

**Published:** 2016-06-06

**Authors:** Qingbo Li, Chuanying Wang, Yanqing Huo, Zhiwei Jia, Xiqian Wang

**Affiliations:** Department of Orthopaedic Trauma, The Second Hospital of Shandong University, Jinan, People’s Republic of China; Department of Rehabilitation, The Second Affiliated Hospital of Shandong University of Traditional Chinese Medicine, No.1 Jingba Road, Jinan, 250001 People’s Republic of China; Department of Orthopaedics, The 306th Hospital of People’s Liberation Army, Beijing, People’s Republic of China

**Keywords:** Achilles tendon rupture, Minimally invasive surgery, Open surgery, Systematic review, Meta-analysis

## Abstract

**Background:**

A number of meta-analyses have been carried out to evaluate the effects of minimally invasive surgery (MIS) versus open surgery (OS) for acute Achilles tendon rupture. However, discordant findings were seen in these meta-analyses. The present study, performing a systematic review of overlapping meta-analyses regarding MIS versus OS of acute Achilles tendon rupture, aimed to assist decision-makers interpret and choose among conflicting meta-analyses, as well as to offer treatment recommendations based on current best evidence.

**Methods:**

The literature search was performed to identify systematic reviews comparing MIS with OS for Achilles tendon rupture. Meta-analyses only comprising randomized controlled trials (RCTs) were included. Two authors individually evaluated the quality of meta-analysis and extracted data. The Jadad decision algorithm was conducted to ascertain which meta-analysis offered the best evidence.

**Results:**

A total of four meta-analyses was included. All these meta-analyses comprised RCTs or quasi-RCTs and were determined as Level-II evidence. The scores of the Assessment of Multiple Systematic Reviews (AMSTAR) ranged from 7 to 10 (median 9.5). The Jadad algorithm indicated that the best meta-analysis should be chosen according to the search strategies and application of selection. A high-quality meta-analysis with more RCTs was chosen, which suggested that there was no statistically significant difference between MIS and OS regarding rerupture rate, tissue adhesion, sural nerve injury, deep infection, and deep vein thrombosis. However, MIS could decrease superficial infection rate, and had a better patient satisfaction for good to excellent outcomes in comparison to OS.

**Conclusions:**

Based on the best available evidence, MIS may be superior to OS for treating acute Achilles tendon rupture. However, due to some limitations, this should be cautiously interpreted, and further high-quality studies are needed.

The article "Minimally invasive versus open surgery for acute Achilles tendon rupture: a systematic review of overlapping meta-analyses" was retracted in 2018. Reasons: plagiarism; overlap with other authors' work.

## Background

Acute Achilles tendon ruptures are frequent traumatic injuries with considerable morbidity [1, 2]. It mainly occurs in male individuals during sports activities, such as tennis, badminton, soccer, and basketball [1, 3]. The prevalence of Achilles tendon rupture is 18 per 100,000 per year and is still increasing because of a rise in the number of populations participating in sport activities [2]. Achilles tendon rupture can be treated by nonsurgical or surgical [4]. The majority of surgeons choose surgical repair for Achilles tendon rupture, because nonsurgical treatment is associated with a high risk of rerupture. In general, surgical treatments for Achilles tendon rupture include minimally invasive surgery (MIS) and open surgery (OS). Although surgical strategies have a rapid progress in recent years, the optimal surgical intervention for acute Achilles tendon ruptures is debatable [5–7].

Several randomized clinical trials (RCTs) comparing MIS with OS for Achilles tendon ruptures have been performed. However, their findings are conflicting [8–13]. In addition, although many meta-analyses of RCTs, representing the best evidence, have been published to compare these two procedures for treating acute Achilles tendon rupture, these overlapping meta-analyses also showed discordant findings [14–17]. These inconsistent findings have resulted in uncertainty for decision-makers with respect to the surgical interventions of Achilles tendon rupture.

In recent years, systematic reviews of overlapping meta-analyses have been reported in many medical fields [18–21]. These studies help to select the best evidence for decision-making by evaluating the overlapping meta-analyses on certain topic [22]. However, to our knowledge, there is no systematic review of overlapping meta-analyses investigating the relative effects between MIS and OS for Achilles tendon rupture. Therefore, the present study aimed to carry out a systematic review of overlapping meta-analyses regarding MIS versus OS for acute Achilles tendon rupture, to assist decision-makers in selecting among conflicting meta-analyses, and to offer intervention recommendations according to the best evidence.

## Methods

This study was performed following the Preferred Reporting Items for Systematic Reviews and Meta-Analysis (PRISMA) statement [23]. The design of this study was based on previous similar publications [18–21].

### Literature search

On August 10, 2015, the databases of PubMed, Embase, and Cochrane Library were systematically retrieved. The keywords were used, including Achilles, systematic review, and meta-analysis. The search strategy was independently conducted by two authors, with the restriction of English language. The references of the included studies were also checked to find possible meta-analyses. The titles and abstracts were first reviewed, and the full texts were acquired if the information was not enough. Disagreements were settled by discussion.

The article "Minimally invasive versus open surgery for acute Achilles tendon rupture: a systematic review of overlapping meta-analyses" was retracted in 2018. Reasons: plagiarism; overlap with other authors' work.

### Eligibility criteria

The inclusion criteria were as follows: (1) comparing MIS with OS for acute Achilles tendon rupture, (2) a meta-analysis only comprising RCTs, and (3) at least one outcome, such as rerupture rate and functional outcome. The narrative review, meetings abstract, correspondence, meta-analysis comprising non-RCTs, and systematic review without meta-analysis conducted were excluded.

### Data extraction

The following data was independently extracted by two authors: first author, year of publications, databases for search, primary study design, the number of RCTs, *I*^2^ statistic value, and outcomes. Disagreements between the two authors were resolved by discussion.

### Quality evaluation

The quality of meta-analysis was evaluated by the Oxford Levels of Evidence [24] and the Assessment of Multiple Systematic Reviews (AMSTAR) instrument [25]. AMSTAR is a methodological assessment with good reliability, validity, and responsibility [26, 27]. It is widely used to evaluate the quality of meta-analysis [20, 21]. The meta-analysis quality was individually evaluated by two authors. Disagreements between authors were settled by discussion.

### Application of the Jadad decision algorithm

The Jadad decision algorithm was used to investigate the origin of inconsistence among systematic reviews, comprising medical question, eligibility criteria, data extraction, quality evaluation, data synthesis, and statistical analysis [22]. It has been widely conducted to offer treatment recommendations among meta-analyses with discordant conclusions [18–21]. This algorithm was independently applied by three authors, who reached a consensus regarding which meta-analysis offered the best evidence.

## Results

### Literature search

A flow chart of the study selection is depicted in Fig. 1. A total of 1382 titles were found from the literature source. Four meta-analyses met the inclusion criteria. The characteristics of these included meta-analyses are listed in Table 1. These studies were published between 2005 and 2012. Table 2 shows that the primary studies (from 2 to 6) of the meta-analyses were published between 1997 and 2009.

**Fig. 1:** The flow chart of study selection

**Table 1:** The characteristics of the included studies

First author	Year	Journal	Date of last literature search	No. of included RCTs
Khan RJ	2005	The Journal of Bone and Joint Surgery, American Volume	NA	2
Khan RJ	2010	Cochrane Database of Systematic Reviews	July 2009	4
McMahon SE	2011	Foot and Ankle Surgery	March 2010	6
Jones MP	2012	The Journal of Bone and Joint Surgery American Volume	NA	4

*RCTs* randomized clinical trials, *NA* not available

The article "Minimally invasive versus open surgery for acute Achilles tendon rupture: a systematic review of overlapping meta-analyses" was retracted in 2018. Reasons: plagiarism; overlap with other authors' work.

**Table 2:** Primary studies included in meta-analyses

First author (Year)	Schroeder D (1997)	Majewski M (2000)	Lim J (2001)	Gigante A (2008)	Aktas S (2009)	Valencia AJA (2009)
Khan RJ (2005)	+		+			
Khan RJ (2010)	+		+	+	+	
McMahon SE (2011)	+	+	+	+	+	+
Jones MP (2012)	+		+	+	+	

### Search methodology

All included meta-analyses had no language restriction. The databases of MEDLINE, Embase, and CINAHL were searched in all meta-analyses, and whether PubMed and Cochrane Library were included in search strategy was heterogenous. Search methodology used in the included meta-analyses is shown in Table 3.

**Table 3:** Search methodology of the included studies

First author (year)	Restriction of publication language	Restriction of publication status	Search database					
			PubMed	MEDLINE	Embase	Cochrane Library	CINAHL	Others
Khan RJ (2005)	No	No		+	+	+	+	+
Khan RJ (2010)	No	No		+	+	+	+	+
McMahon SE (2011)	No	No	+	+	+		+	+
Jones MP (2012)	No	No		+	+	+	+	+

### Quality evaluation

All meta-analyses comprised RCTs or quasi-RCTs and were determined as Level-II evidence according to the Oxford Levels of Evidence (Table 4). The AMSTAR scores for the included meta-analyses are listed in Table 5, ranging from 7 to 10 (median 9.5). Two Cochrane reviews with 10 scores of AMSTAR were the highest-quality studies.

**Table 4:** Methodological information of the included studies

First author (year)	Design of included studies	Level of evidence	Software	GRADE use	Sensitivity analysis
Khan RJ (2005)	RCT or quasi-RCT	Level II	NA	No	No
Khan RJ (2010)	RCT or quasi-RCT	Level II	NA	No	No
McMahon SE (2011)	RCT or quasi-RCT	Level II	RevMan	No	No
Jones MP (2012)	RCT or quasi-RCT	Level II	NA	No	No

*RCT* randomized controlled trial, *NA* not available

**Table 5:** AMSTAR scores of the included studies

Items	Khan RJ (2005)	Khan RJ (2010)	McMahon SE (2011)	Jones MP (2012)
1. Was an a priori design provided?	0	1	0	1
2. Was there duplicate study selection and data extraction?	1	1	1	1
3. Was a comprehensive literature search performed?	1	1	1	1
4. Was the status of publication (i.e., grey literature) used as an inclusion criterion?	0	1	1	1
5. Was a list of studies (included and excluded) provided?	1	1	0	1
6. Were the characteristics of the included studies provided?	0	1	1	1
7. Was the scientific quality of the included studies assessed and documented?	1	1	1	1
8. Was the scientific quality of the included studies used appropriately in formulating conclusions?	1	1	1	1
9. Were the methods used to combine the findings of studies appropriate?	1	1	1	1
10. Was the likelihood of publication bias assessed?	0	0	1	0
11. Was the conflict of interest stated?	1	1	1	1
Total scores	7	10	9	10

The article "Minimally invasive versus open surgery for acute Achilles tendon rupture: a systematic review of overlapping meta-analyses" was retracted in 2018. Reasons: plagiarism; overlap with other authors' work.

### Heterogeneity assessment

The *I*^2^ statistic value, as a measurement tool for investigating the interstudy variability, was used to evaluate the heterogeneity among primary studies in each meta-analysis (Table 6). None of the included studies performed sensitivity analyses (Table 4). The *I*^2^ statistic values of all included meta-analyses are listed in Table 6. The heterogeneities are acceptable for most outcomes.

**Table 6:** *I* ^2^ statistic value of each variable in each meta-analysis

Items	Khan RJ (2005)	Khan RJ (2010)	McMahon SE (2011)	Jones MP (2012)
Rerupture	NA	0.0 %	0 %	NA
Complications excluding rerupture	0.0 %			
Superficial infection		0.0 %	0 %	
Deep infection		0.0 %	0 %	
Wound infection	0.0 %	0.0 %		0 %
Deep vein thrombosis		0.0 %	0 %	
Delayed wound healing		NA		
Ankle stiffness		NA		
Disturbing scar/wound puckering		64 %		
Adhesions		0.0 %	0 %	
Failed repair (tendon elongation)		NA		
Hematoma		NA		
Keloid formation		NA		
Sural nerve injury		NA	0 %	
Tendinopathy		NA		
SF-12 physical component		NA		
Subjective outcomes (good to excellent)			0 %	
Subjective outcomes (fair)			76 %	

*NA* not available

### Results of the Jadad decision algorithm

Which meta-analysis offered the best available evidence among the four included meta-analyses was investigated following the Jadad decision algorithm [22]. The meta-analysis results of the included studies are depicted in Fig. 2. Based on that the included studies investigated the same question, did not comprise the same studies, and that the eligibility criteria were similar, the Jadad decision algorithm indicated that the best available evidence should be chosen according to the search strategies and application of selection (Fig. 3). Therefore, a high-quality study with more RCTs was selected. This study demonstrated that MIS for Achilles tendon rupture provided a lower superficial infection rate and a better subjective patient satisfaction, while not raising the risk of rerupture, tissue adhesion, sural nerve injury, deep infection, and deep vein thrombosis in comparison to OS.

**Fig. 2:** Results of the included meta-analyses

**Fig. 3:** The flow chart of the Jadad decision algorithm

## Discussion

Achilles tendon ruptures can be treated surgically using either MIS or OS [3, 28–30]. In recent years, multiple meta-analyses have been conducted to assess the difference regarding MIS versus OS. However, discordant results were observed among these meta-analyses [14–17], which complicated decision-makers. To solve this problem, systematic reviews of overlapping meta-analyses are increasingly published in medical fields [18–21]. To our knowledge, this is the first systematic review of overlapping meta-analyses on the topic of MIS versus OS for acute Achilles tendon ruptures. In this study, four meta-analyses were included using a systematic literature review. Based on the Jadad decision algorithm, a high-quality meta-analysis with more RCTs was selected as the current best available evidence [14].

The article "Minimally invasive versus open surgery for acute Achilles tendon rupture: a systematic review of overlapping meta-analyses" was retracted in 2018. Reasons: plagiarism; overlap with other authors' work.

We found that most of the meta-analyses comprehensively conducted the literature search within a similar period, but they did not include the same primary trials, and did not provide the same conclusion on the surgical intervention for acute Achilles tendon rupture [14–17]. This phenomenon can be attributed to multiple factors, including the clinical question, study selection and inclusion, data extraction, quality evaluation, assessment of the ability to combine studies, and statistical methods for data pooling [22]. A decision algorithm, which was adopted in this study, was designed to choose the high-quality level of evidence from currently discordant systematic reviews [22]. This tool was widely used to find the best available evidence among overlapping systematic reviews [18–21].

In this study, the meta-analysis by McMahon et al. [14] was selected according to the Jadad decision algorithm. Their study demonstrated that there were no differences between MIS and OS with respect to rerupture, deep infection, deep vein thrombosis, adhesions, sural nerve injury, and subjective outcomes (fair). However, MIS was superior to OS in superficial infection and subjective outcomes (good to excellent). In other words, when comparing with OS, MIS could decrease the incidence of superficial infection and could improve subjective patient satisfaction, while not raising the risk of rerupture. Therefore, the best available evidence suggests that MIS may be superior to OS for the treatment of acute Achilles tendon rupture. This conclusion should be cautiously interpreted and confirmed by further well-designed RCTs due to the small sample size of the selected meta-analysis.

There are several limitations in this study. First, the literature search was limited to English papers. Non-English literature could not be included in this systematic review, despite that multiple databases were searched. Second, in order to get the best available evidence, only meta-analyses of RCTs were comprised. Nevertheless, all the included studies were Level-II evidence. Therefore, this systematic review could not offer treatment recommendations based on Level-I evidence.

The article "Minimally invasive versus open surgery for acute Achilles tendon rupture: a systematic review of overlapping meta-analyses" was retracted in 2018. Reasons: plagiarism; overlap with other authors' work.

## Conclusions

Based on the systematic review of overlapping meta-analyses regarding MIS versus OS for acute Achilles tendon rupture, MIS may be superior to OS for treating acute Achilles tendon rupture. However, large and high-quality RCTs are still needed to confirm this finding due to the limitations of the current evidence.

## Abbreviations

*AMSTAR* Assessment Of Multiple Systematic Reviews, *MIS* minimally invasive surgery, *OS* open surgery, PRISMA, Preferred Reporting Items For Systematic Reviews And Meta-Analysis, *RCTs* randomized controlled trials
